The article "Variability and Patterning in Permanent Tooth Dimensions among Four Ethnic Groups from the North-eastern States of India" was published in 2022. Journal: Biomed Res Int.

# Variability and Patterning in Permanent Tooth Dimensions among Four Ethnic Groups from the North-eastern States of India

**DOI:** 10.1155/2022/4733611

**Published:** 2022-09-13

**Authors:** Plabita Majumder, Putul Mahanta, Chandana Kalita, Madhab Ch. Rajbangshi, Dipanjal Saikia, Ranjumoni Konwar, Bharati Basumatari, N. Sherin

**Affiliations:** ^1^Dentistry, Tezpur Medical College and Hospital, Tezpur, 784010 Assam, India; ^2^Forensic Medicine and Toxicology, Assam Medical College, 786002, Dibrugarh, Assam, India; ^3^Conservative Dentistry and Endodontics, Govt Dental College, 786002, Dibrugarh, Assam, India; ^4^Surgery, Tezpur Medical College and Hospital, Tezpur, 784010 Assam, India; ^5^Dentistry, Assam Medical College and Hospital, Dibrugarh, 786002 Assam, India; ^6^Radiology, Gauhati Medical College and Hospital, Guwahati, 32 Assam, India; ^7^Radiology, Fakhruddin Ali Ahmed Medical College and Hospital, Barpeta, 781301 Assam, India; ^8^Govt Dental College, 786002, Dibrugarh, Assam, India

## Abstract

**Methods:**

The study was a comparative cross-sectional study among four different ethnic groups of North-east India among the age group of 20-30 years. Dimensions of the maxillary and mandibular teeth were measured with a digital Vernier calliper using the dental casts of 50 male and 50 female subjects from each of the four ethnic groups under study. The data were statistically analyzed using a Student's *t*-test and one-way analysis of variance. Statistical significance was set at *p* < 0.05.

**Results:**

The tooth dimensions of all four ethnic groups were significantly lower than the standard values except for the MD dimension of the maxillary second molars of the Singpho group (9.13 mm vs. 9.0 mm); mandibular central incisors of the Meitei group (5.01 mm vs. 5.0 mm); and mandibular lateral incisors of the Meitei, Ao, and Singpho groups (>standard value of 5.5 mm) and BL dimension of the mandibular first premolars of the Meitei and Ao groups (>standard value of 7.5 mm); mandibular second premolars of the Meitei and Singpho groups (>standard value of 8.0 mm); and mandibular second molars of the Ao group (10.04 mm vs. 10.0 mm). In some instances, the comparative analysis revealed group variations in different tooth dimensions among the four ethnic groups (*p* < 0.05).

**Conclusion:**

Variations were observed in the tooth dimensions among the four ethnic groups and within the same population. Unlike other parts of India, the North-eastern population belongs to a distinct ethnic race of indigenous people of East Asia, Southeast Asia, and the Arctic region of North America. Hence, population-specific data for India's North-eastern region are necessary for forensic odontology, dental anthropology, routine dental practice, and effective treatment planning.

The article "Variability and Patterning in Permanent Tooth Dimensions among Four Ethnic Groups from the North-eastern States of India" was published in 2022. Journal: Biomed Res Int.

## 1. Introduction

Physical anthropologists, human biologists, and geneticists universally agree that all humans are descendants of the same species (Homo sapiens) and, thus, share a common ancestry. However, there are several different human groups. Individual variations within a population or the distinction between human groups referred to as races are caused by genetic variation and environmental effects. Determination of ethnicity is the most controversial issue in identifying unknown individuals, and it is difficult to associate any specific anatomical trait with a certain race. However, careful physical, skeletal, and dental assessments may assist in establishing an individual's racial identity [1].

Teeth can reveal necessary information about the nature and scope of diversity among human populations. Different populations within the same demographic area have shown differences in dental crown size [2]. Variations in tooth form are widespread in permanent dentition and are crucial for ethnic, forensic, and anthropological purposes [3]. Heredity, ethnicity, sex, and evolutionary trends substantially influence the variations in tooth size among different groups and ethnicities [3]. These morphometric traits of the teeth can be used to assess a person's age, sex, race, socioeconomic status, work habits, oral and systemic health, occupation, and nutritional quality [4]. Odontometry is an anthropological science that dates to the first half of the eighteenth century and is used to discern different groups and populations based on their dental features [5]. In forensic dentistry, odontometry plays a significant role in identifying individuals, and it also plays a role in clinical dentistry for treatment planning.

India is a vast country with a diverse population, including many races and ethnicities. Thus, there is a high possibility of variable tooth dimensions among individuals, necessitating the creation of a region-specific odontometric database to identify individuals and provide high-quality population-specific dental treatment. Population from India's North-eastern states has a pure genetic pool, with over 60–70% of the population being tribal and belonging to the indigenous peoples of East Asia, Southeast Asia, and the Arctic region of North America. Information regarding the tooth dimensions of this population is scarce, and no odontometric studies have been performed in this region. Therefore, the present odontometric survey included four ethnic groups in North-eastern India: Miching of Assam, Singpho of Arunachal Pradesh, Ao of Nagaland, and Meitei of Manipur.

The article "Variability and Patterning in Permanent Tooth Dimensions among Four Ethnic Groups from the North-eastern States of India" was published in 2022. Journal: Biomed Res Int.

The study's research question was whether any differences in variability and patterning in dental crown sizes exist among the four ethnic groups of Northeast India. The study aimed to evaluate the mesiodistal (MD), buccolingual (BL), and cervico-incisal (C-I) tooth dimensions using dental casts and to compare the variability and patterning of tooth dimensions with existing standard data among the groups under study.

## 2. Materials and Methods

The present comparative cross-sectional study was conducted at the Department of Oral Pathology and Microbiology, Kothiwal Dental College and Research Center, Moradabad. The study included individuals aged 20–30 years who had a complete set of healthy teeth and gingiva up to the second molars. Individuals with significant loss of tooth substance due to attrition, caries, or restoration or those who had undergone orthodontic treatment were excluded. An oral examination was performed before inclusion. Informed consent was obtained from all participants. The dimensions of central incisors (CI), lateral incisors (LI), canines (C), first premolars (PM1), second premolars (PM2), first molars (M1), and second molars (M2) were measured. The data were recorded on a separately prepared, custom-made record sheet. The study was approved by the institutional ethical review board (vide letter no. KDCRC/IERB/OP/2014/23).

### 2.1. Study Population and Samples

The present study included four ethnic groups in North-eastern India: Miching (Assam), Meitei (Manipur), Ao (Nagaland), and Singpho (Arunachal Pradesh). Miching is Assam's second most populous scheduled tribe. These individuals are all blood-brothers due to various social constraints in their marital connections. Nagaland's Ao is the dominant ethnic group in the dialect. Meitei is the most populous ethnic group in Manipur, accounting for more than 60% of the state's population. The Singpho community is a member of the Burmese Kachin tribe inhabiting Arunachal Pradesh's Lohit and Changlang districts.

Using simple random sampling, we selected 50 male and 50 female subjects from each of the four ethnic groups (age: 20–30 years). The samples were collected from the native place of all those dominated areas of various ethnic groups. Measurements were performed on the dental casts of the participants using a digital Vernier calliper to determine the tooth dimensions.

### 2.2. Measurement of Tooth Dimensions

Irreversible hydrocolloid impressions of all participants' maxillary and mandibular dentitions were made using appropriate perforated trays [6]. To avoid model distortion, impressions were promptly poured with high-quality dental stone [7]. The MD dimension of the crown of the tooth was determined by measuring the most significant distance between the approximated surface of the crown using a sliding calliper with pointed tips held parallel to the occlusal and vestibular surfaces of the crown. Holding the callipers perpendicular to the MD axis of the tooth, the largest BL measurement was considered the BL dimension of the crown. The C-I dimension of the crown was measured from the crest of curvature at the cementoenamel junction to the incisal edge or the buccal cusp tip.

The article "Variability and Patterning in Permanent Tooth Dimensions among Four Ethnic Groups from the North-eastern States of India" was published in 2022. Journal: Biomed Res Int.

### 2.3. Statistical analysis

The data were statistically analyzed using IBM SPSS Statistics (version 20; IBM Corp., Armonk, NY, USA) and compared with the existing standard odontometric data, as suggested in Wheeler's Dental Anatomy, Physiology, and Occlusion [8]. Quantitative variables were presented as mean ± standard deviation. Differences between mean values were analyzed using the Student's *t*-test and one-way analysis of variance with posthoc tests or their nonparametric complements depending on the normality of the data. The normality of the data was tested using Kolmogorov-Smirnov (K-S) test. Statistical significance was set at a *p* < 0.05.

## 3. Results

Altogether, 5600 tooth samples were assessed for different tooth dimensions using the dental casts of 400 participants (50 males and 50 females from each of the four ethnic groups). Since the data had a normal distribution (*p* value for the K − S test > 0.05 for all the tooth dimensions for the four ethnic groups), the mean tooth dimensions were compared using a one-way analysis of variance with posthoc analysis.

The mean MD dimensions of all anterior maxillary teeth were significantly lower (*p* < 0.05) than the standard values except for the maxillary LI (mean: 6.28 mm) and maxillary C (mean: 7.17 mm) of the Singpho group. The mean MD dimension of the maxillary CI in the Meitei group and that of the maxillary LI in the Ao group were substantially lower than the standard value. Among the posterior maxillary teeth, the MD dimension of the maxillary M1 of the Miching group was significantly different from that of the other three groups. Similarly, the mean MD dimensions of all the mandibular anterior teeth were lower than the corresponding standard values except for the MD dimension of the LI of the Meitei, Ao, and Singpho groups. The Miching group exhibited the smallest mean MD dimensions of the mandibular CI and LI. Moreover, the four groups differed substantially in the MD dimension of the mandibular C. The Singpho group exhibited the largest mean MD dimensions of the mandibular CI and C. Furthermore, the MD dimensions of the mandibular posterior teeth were significantly lower in all four ethnic groups compared to the standard orthodontic data (Table 1).

The article "Variability and Patterning in Permanent Tooth Dimensions among Four Ethnic Groups from the North-eastern States of India" was published in 2022. Journal: Biomed Res Int.

Among the anterior maxillary teeth, BL dimensions of all four ethnic groups were significantly lower than the standard values (*p* < 0.05) except for the maxillary LI of the Miching and Meitei groups and the maxillary C of the Singpho group. Moreover, comparative analyses of Miching vs. Ao, Miching vs. Singpho, and Meitei vs. Ao for the maxillary CI and Miching vs. Ao, Miching vs. Singpho, and Meitei vs. Singpho for the maxillary LI exhibited significant (*p* < 0.05) differences in the mean BL dimensions. Among the posterior maxillary teeth, the mean BL dimensions were significantly lower (*p* < 0.05) compared with the standard values except for the PM1 in the Meitei and Singpho groups and PM2 in the Singpho group, and M1 in the Miching and Ao groups. Significant variability in the BL dimension of the mandibular CI was observed when the Miching group was compared with the Ao and Singpho groups. Significant variability in the BL dimension of the mandibular C was observed when the Miching group was compared with the other three groups. The Ao group exhibited the most significant dimensions of the mandibular PM1. The Miching and Ao groups had smaller mean BL dimensions of the mandibular PM2 compared to the standard values. All four groups exhibited smaller mean BL dimensions of the mandibular M1 compared to the standard values. The difference was not statistically significant except in the case of the Miching group. The mean BL dimensions of the mandibular M2 in all ethnic groups were significantly smaller than the standard values except for the Ao group (mean: 10.05 mm). The Miching group exhibited the lowest mean BL dimensions of the M2 in both jaws (Table 2).

The C-I dimensions of all teeth of all four ethnic groups were significantly lower than the standard values. The C-I dimension of the maxillary CI showed statistically significant variability (*p* < 0.05) in the comparative analysis of Miching vs Ao, Miching vs. Singpho, and Meitei vs. Ao. Similarly, the mean C-I dimension of the maxillary C in the Miching group (mean: 7.85 mm) differed significantly from that in other groups. The Miching group also exhibited the smallest C-I dimension of the maxillary PM2 (mean: 5.47 mm). In addition, the mean C-I dimension of the maxillary M2 differed substantially between the Meitei and Singpho groups. Comparative data analysis of Miching vs. Ao and Meitei vs. Ao for the mandibular LI and Miching vs. Ao for the mandibular C revealed a substantial difference in mean C-I dimensions (*p* < 0.05). Moreover, the mean C-I dimensions of the mandibular PM1 differed substantially in the comparative analysis of Miching vs. Meitei, Miching vs. Ao, and Meitei vs. Singpho groups. The mean C-I dimension of the mandibular PM2 differed considerably in the comparative analysis of Miching vs. Meitei and Miching vs. Singpho groups. In all four ethnic groups, the between-group analysis revealed a significant variation in the mean C-I dimension of the mandibular M2 (Table 3).

The article "Variability and Patterning in Permanent Tooth Dimensions among Four Ethnic Groups from the North-eastern States of India" was published in 2022. Journal: Biomed Res Int.

## 4. Discussion

The present comparative study was undertaken to evaluate the mesiodistal (MD), buccolingual (BL), and cervico-incisal (C-I) tooth dimensions of four ethnic groups of North-eastern India using dental casts and to compare the variability and patterning of tooth dimensions with existing standard data and among the four groups.

Except for the maxillary M2 in the Singpho group and the mandibular LI in the Meitei, Ao, and Singpho groups, the MD dimensions of all teeth of the four ethnic groups were lower than the standard values. These findings are consistent with previous research conducted among the indigenous peoples of East Asia, Southeast Asia, and the Arctic region of North America [9–11]. Moreover, the results of multiple additional studies corroborate the present findings, implying that different communities have distinct tooth morphometric parameters, necessitating the compilation of population-specific data [4, 12, 13] . However, contrary to our results, the MD dimensions were larger than the standard values in some studies conducted in India [14–16] and the rest of the world [17–21]. These differences could be because our study sample comprised distinct ethnic groups of indigenous peoples of East Asia, Southeast Asia, and the Arctic region of North America.

Except for the mean BL dimension of the PM2 in the Meitei and Singpho ethnic groups, the mean BL dimensions of the teeth in both jaws were smaller when compared with the standard odontometric data. Similar findings have been reported in previous research conducted among the indigenous peoples of East Asia, Southeast Asia, and the Arctic region of North America [9–11]. Another study found lower BL dimensions among different study populations, indicating a drop in the BL dimension when the standard value was not specific to the indigenous peoples of East Asia, Southeast Asia, and the Arctic region of North America [4]. However, a few investigations from North India [15] and South India [16] reported that the BL dimensions were higher than the standard values, contradicting the present study's findings. Another study involving Colombian Caucasian mestizos reported that the BL dimension was much higher than the standard odontometric value [18]. This difference can be linked to a specific genetic trait or the average height/build of the population.

The article "Variability and Patterning in Permanent Tooth Dimensions among Four Ethnic Groups from the North-eastern States of India" was published in 2022. Journal: Biomed Res Int.

The present study observed significantly lower C-I dimensions in all ethnic groups compared to the standard values. Very few studies have measured the C-I dimension on the dental cast since the true C-I dimension of a tooth should be assessed in extracted teeth. However, a Turkish survey [22] revealed a decrease in the anterior teeth C-I dimension compared to the standard value, which is consistent with our findings. Lower C-I dimensions in the present study may be due to the tooth's lower MD and BL dimensions compared with the standard data. Further studies, including larger sample sizes and various populations from North-eastern India, may ascertain the C-I dimensions, adding to the accuracy of tribe-specific identification of individuals.

Variations in tooth dimensions among different populations might be attributed to the differences in average height, weight, body build, eating habits, race, gender, hereditary factors, and environmental factors [20]. The lower tooth size observed in our study sample could be attributed to the overall below-average height/build of the indigenous peoples of East Asia, Southeast Asia, and the Arctic region of North America population. Furthermore, the typical dietary habits in these communities may be linked to lower tooth size. Most of the ethnic populations in this region utilize earthenware to prepare food into liquid or ‘semiliquid' consistency. Thus, due to the reduced chewing requirement, there might be a relaxation in the intensity of selection forces for maintaining tooth size [23].

Brook et al. reported differences in the crown size patterns between different populations, with notably greater size variation among later-forming teeth [24]. Additional tooth traits such as the cusp of Carabelli, shovel-shaped incisors, and premolars with multiple cusps can also help determine ancestry [25]. A parabolic arch with larger incisors and canines, smaller premolars, and larger molars, especially in the lower arch; a lower prevalence of the Carabelli's trait; and a higher prevalence of shovel incisors are signs of the indigenous peoples of East Asia, Southeast Asia, and the Arctic region of North America [26, 27]. In the present study, we observed large incisors and canines, small premolars, and large molars, which are common features of the dentition of those indigenous peoples of East Asia, Southeast Asia, and the Arctic region of North America, particularly in the lower arch [1]. A study involving North Indian and North-eastern Indian populations revealed that most permanent teeth except the maxillary CI, maxillary PM1, and maxillary M2 in North-eastern Indians exhibited BL dimensional variations. These findings partially agree with our study's results [28].

The article "Variability and Patterning in Permanent Tooth Dimensions among Four Ethnic Groups from the North-eastern States of India" was published in 2022. Journal: Biomed Res Int.

Among the three major racial groups of people having European ancestry; the indigenous peoples of East Asia, Southeast Asia, the Arctic region of North America and the indigenous peoples of central and southern Africa, each race has unique characteristics related to dentition.

However, due to racial hybridization worldwide, assigning a racial identity to an unknown individual cannot be based exclusively on dental morphological features. Even though the dental morphological features of the three major races have merged, some traits are dominant in some ethnic groups [29]. Due to the wide range of morphological traits and their forms, human dental traits are helpful diagnostic tools for anthropological studies to identify and describe different ethnic groups [30]. The results of the present study helped establish the idea of regional or ethnic variation in dental morphometry by demonstrating variations in tooth dimensions among four ethnic groups from North-eastern India compared with the standard values. Even within the same population, the variability and uniqueness of tooth dimensions observed in individuals belonging to the four ethnic groups in North-eastern India indicate the need for population-specific odontometric data to identify individuals belonging to these ethnicities.

### 4.1. Limitations

The present study included only four ethnic groups in North-eastern India. However, the study region has vast ethnic and tribal diversity, and a more detailed study including tribal and nontribal populations may help generalize the present study results.

## 5. Conclusions

Most of the teeth in our study population exhibited lower MD, BL, and C-I dimensions than the standard values, with variability among different ethnic groups and even within the same group. The differences in tooth dimensions among the four ethnic groups demonstrate the need for population-specific odontometric data for these distinct communities.

## Figures and Tables

**Table 1:** Mesiodistal dimensions of permanent teeth among the four ethnic groups.

Tooth	Arch	Mean ± standard deviation					*p* value^#^
		Miching	Meitei	Ao	Singpho	Standard	
CI	Maxilla	8.09 (0.4)	7.66 (0.08)	8.04 (0.07)	7.95 (0.09)	8.5 (0.0)	<0.001
	Mandible	4.52 (0.29)	5.01 (0.79)	4.89 (0.34)	4.86 (0.50)	5.0 (0.0)	<0.001
LI	Maxilla	6.23 (0.48)	6.13 (0.43)	5.77 (0.35)	6.28 (0.62)	6.5 (0.0)	<0.001
	Mandible	5.18 (0.51)	5.56 (0.52)	5.55 (0.52)	5.67 (0.49)	5.5 (0.0)	<0.001
C	Maxilla	6.87 (0.44)	7.14 (0.39)	6.97 (0.51)	7.17 (0.94)	7.5 (0.0)	<0.001
	Mandible	6.23 (0.534)	6.39 (0.58)	6.17 (0.47)	6.66 (0.73)	7.0 (0.0)	<0.001
PM1	Maxilla	6.59 (0.45)	6.57 (0.69)	6.64 (0.40)	6.37 (0.39)	7.0 (0.0)	<0.001
	Mandible	6.45 (0.40)	6.61 (0.42)	6.44 (0.35)	6.45 (0.56)	7.0 (0.0)	<0.001
PM2	Maxilla	5.91 (0.46)	5.96 (0.75)	5.83 (0.48)	5.82 (0.59)	7.0 (0.0)	<0.001
	Mandible	6.02 (0.28)	6.12 (0.64)	6.16 (0.33)	6.11 (0.44)	7.0 (0.0)	<0.001
M1	Maxilla	9.87 (0.71)	9.23 (0.25)	9.23 (0.53)	9.52 (0.59)	10.0 (0.0)	<0.001
	Mandible	10.32 (0.45)	10.47 (0.79)	10.28 (0.55)	10.13 (0.71)	11.0 (0.0)	<0.001
M2	Maxilla	8.95 (0.49)	8.92 (0.82)	8.82 (0.51)	9.13 (0.47)	9.0 (0.0)	0.119
	Mandible	9.30 (0.69)	9.46 (0.78)	9.24 (0.39)	9.31 (0.49)	10.5 (0.0)	<0.001

^#^ *p* value for one-way ANOVA.

The article "Variability and Patterning in Permanent Tooth Dimensions among Four Ethnic Groups from the North-eastern States of India" was published in 2022. Journal: Biomed Res Int.

**Table 2:** Comparison of buccolingual dimensions of permanent teeth among the four ethnic groups.

Tooth	Arch	Mean ± standard deviation					*p* value^#^
		Miching	Meitei	Ao	Singpho	Standard	
CI	Maxilla	6.06 (0.51)	6.25 (0.57)	6.71 (0.62)	6.45 (0.31)	7.00 (0.0)	<0.001
	Mandible	5.23 (0.51)	5.64 (0.62)	5.57 (0.47)	5.64 (0.59)	6.00 (0.0)	<0.001
LI	Maxilla	5.32 (0.50)	5.52 (0.57)	5.73 (0.81)	5.86 (0.54)	6.00 (0.0)	<0.001
	Mandible	5.67 (0.43)	5.74 (0.58)	5.72 (0.60)	5.82 (0.52)	6.5 (0.0)	<0.001
C	Maxilla	7.00 (0.27)	7.52 (0.76)	7.47 (0.52)	7.29 (0.39)	8.00 (0.0)	<0.001
	Mandible	6.47 (0.47)	6.95 (0.71)	7.11 (0.40)	6.81 (0.50)	7.5 (0.0)	<0.001
PM1	Maxilla	8.64 (0.47)	8.48 (1.17)	8.44 (0.84)	8.74 (0.43)	9.00 (0.0)	<0.001
	Mandible	7.38 (0.33)	7.59 (0.53)	7.93 (0.68)	7.35 (0.35)	7.5 (0.0)	<0.001
PM2	Maxilla	8.75 (0.51)	8.61 (0.49)	8.59 (0.20)	8.81 (0.38)	9.00 (0.0)	<0.001
	Mandible	7.89 (0.26)	8.12 (0.61)	7.89 (0.40)	8.29 (0.52)	8.0 (0.0)	<0.001
M1	Maxilla	11.03 (0.68)	10.62 (0.57)	10.74 (0.37)	10.62 (0.31)	11.00 (0.0)	<0.001
	Mandible	10.13 (0.55)	9.90 (0.67)	10.24 (0.46)	10.31 (0.35)	10.5 (0.0)	0.006
M2	Maxilla	10.29 (0.69)	10.35 (0.44)	10.65 (0.44)	10.58 (0.57)	11.00 (0.0)	<0.001
	Mandible	9.46 (0.72)	9.84 (0.55)	10.05 (0.35)	9.98 (0.32)	10.0 (0.0)	<0.001

^#^ *p* value for one-way ANOVA.

**Table 3:** Comparison of cervico-incisal dimensions of permanent teeth among the four ethnic groups.

Tooth	Arch	Mean ± standard deviation					*p* value^#^
		Miching	Meitei	Ao	Singpho	Standard	
CI	Maxilla	8.00 (0.74)	8.04 (1.06)	8.57 (0.81)	8.73 (0.74)	10.50 (0.0)	<0.001
	Mandible	7.01 (0.67)	7.18 (1.37)	7.16 (0.45)	7.44 (0.60)	9.5 (0.0)	<0.001
LI	Maxilla	6.96 (0.61)	7.40 (1.15)	7.20 (0.85)	7.33 (0.65)	9.00 (0.0)	<0.001
	Mandible	7.11 (0.90)	6.87 (1.27)	7.64 (1.06)	7.24 (0.30)	9.5 (0.0)	<0.001
C	Maxilla	7.85 (0.50)	8.52 (1.19)	8.35 (0.74)	8.71 (0.62)	10.00 (0.0)	<0.001
	Mandible	7.91 (1.10)	8.45 (1.64)	8.64 (0.68)	8.24 (0.74)	11.0 (0.0)	<0.001
PM1	Maxilla	6.82 (0.38)	7.02 (0.90)	7.14 (0.72)	7.14 (0.55)	8.50 (0.0)	<0.001
	Mandible	7.22 (0.38)	7.61 (0.94)	7.57 (0.51)	7.27 (0.44)	8.5 (0.0)	<0.001
PM2	Maxilla	5.47 (0.75)	5.80 (0.89)	5.94 (0.52)	5.97 (0.57)	8.50 (0.0)	<0.001
	Mandible	5.90 (0.76)	6.30 (0.99)	6.18 (0.51)	6.29 (0.38)	8.0 (0.0)	<0.001
M1	Maxilla	5.50 (0.59)	5.59 (0.78)	5.59 (0.61)	5.61 (0.58)	7.50 (0.0)	<0.001
	Mandible	5.39 (1.17)	5.51 (0.74)	5.49 (0.45)	5.81 (0.43)	7.0 (0.0)	<0.001
M2	Maxilla	5.17 (0.39)	4.87 (0.69)	5.31 (0.73)	5.50 (0.55)	7.00 (0.0)	<0.001
	Mandible	5.39 (1.17)	5.51 (0.74)	5.49 (0.45)	5.81 (0.43)	7.0 (0.0)	<0.001

^#^ *p* value for one-way ANOVA.

The article "Variability and Patterning in Permanent Tooth Dimensions among Four Ethnic Groups from the North-eastern States of India" was published in 2022. Journal: Biomed Res Int.

## Data Availability

Data supporting the findings of this study are available within the article.
